The article "High Throughput Screening for Bioactive Components of Berberis baluchistanica Ahrendt Root and Their Functional Potential Assessment" was published in 2022. Journal: Biomed Res Int.

# High Throughput Screening for Bioactive Components of *Berberis baluchistanica* Ahrendt Root and Their Functional Potential Assessment

**DOI:** 10.1155/2022/1746116

**Published:** 2022-07-26

**Authors:** Zareen Gul, Ali Akbar, Imran Ali, Javed Muhammad, Zia Ur Rehman, Amna Bano, Abdul Samad, Amjad Khan, Samiullah, Saadullah Khan Leghari, Su Hlaing Chein, Ali A. Rabaan

**Affiliations:** ^1^Department of Microbiology, University of Balochistan, Quetta, Balochistan, Pakistan; ^2^Department of Botany, University of Balochistan, Quetta, Balochistan, Pakistan; ^3^Institute of Biochemistry, University of Balochistan, Quetta, Balochistan, Pakistan; ^4^Department of Microbiology, The University of Haripur, Pakistan; ^5^Department of Chemistry, University of Balochistan, Quetta, Balochistan, Pakistan; ^6^Center for Advanced Studies in Vaccinology & Biotechnology (CASVAB), University of Balochistan, Quetta, Pakistan; ^7^Department of Public Health and Nutrition, The University of Haripur, Pakistan; ^8^Spectrum-Sustainable Development Knowledge, Yangon 11111, Myanmar; ^9^Molecular Diagnostic Laboratory Johns Hopkins Aramco Healthcare Dhahran, Saudi Arabia

## Abstract

*Berberis baluchistanica* Ahrendt is a medicinal plant potentially known for the treatment of different diseases. The bioactive, antioxidant, nutritional components, and antimicrobial properties of crude ethanolic root extract of *Berberis baluchistanica* were evaluated in this study. The extract was analyzed for total phenolic, flavonoid, DPPH (2, 2-diphenyl-1-picryl-hydrazyl) scavenging ability, FRAP (ferric reducing antioxidant power), nutritional, and antimicrobial potentials. The alkaloids, tannins, cardiac glycosides, anthraquinones, coumarin, saponins, phenolics, flavonoids, steroids, and terpenoids were confirmed. The extract possessed DPPH radical inhibition with the IC_50_ of 1.125 mg/mL and FRAP % reduction activity with IC_50_ (0.912 mg/mL). Total phenolic 19.897 ± 4.8141 mg GAE/g and flavonoid 12.9876 ± 0.8388 mg QE/g contents were confirmed in the root. The extracts exhibit good antibacterial activity against a broad spectrum of food borne pathogens *Pseudomonas aeruginosa*, *Salmonella typhi*, *Klebsiella pneumoniae*, *Escherichia coli*, and *Staphylococcus aureus*. The highest inhibitory activity was against *Escherichia coli*23.30 ± 1.16 mm and lowest against *Klebsiella pneumoniae*7 ± 0.01 mm. Furthermore, the presence of various phytochemical constituents (plant secondary metabolites) was also confirmed with gas chromatography and mass spectroscopy analysis. Results disclosed the occurrence of more than 70 compounds possessing various medicinal properties supporting the traditional uses of root of *Berberis baluchistanica* in various medical complications indigenously.

The article "High Throughput Screening for Bioactive Components of Berberis baluchistanica Ahrendt Root and Their Functional Potential Assessment" was published in 2022. Journal: Biomed Res Int.

## 1. Introduction

Therapeutic plants have significant positive role in individual and communities health [1, 2]. These plants and their components are traditionally in use for the treatment of many diseases such as fever, cough, internal injury, eye disease, removal of kidney stones, wound healing, rheumatism, and other infections of human beings and livestock [3, 4]. Herbal medicines contain an intricate combination of various significant bioactive components such as alkaloids, polyphenols, flavonoids, terpenoids, minerals, and vitamins. These components have considerable antimicrobial, anti-inflammatory, cytotoxic, and antioxidant potential to reduce free radicals. It decreases the production of lipid peroxidation in human bodies, which are responsible for a variety of human diseases. The herbal medicines containing these phytochemical constituents (plant secondary metabolites) are used as alternate of synthetic drugs which are hazardous for both human and environment [5]. The presence of these bioactive and antioxidant components in plants have increased their therapeutic and nutritional values and overall demand as a folk medicines [1].

The genus Berberis belongs to family Berberidaceae, with 15 genera and 650 species [6]. It is among the primitive angiosperm having great economic and medicinal values [7]. Different phytochemicals such as glycosides, steroids, anthraquinones, anthraquinones, saponins, alkaloids, phlobatannins, tannins, reducing sugars, flavonoids, terpenoids, oleanolic acid, palmatine, and stigmasterol have also been confirmed in Berberis [8]. The antioxidant, antidiabetic, antibacterial, anti-inflammatory, heptoprotective, and hypotensive properties of berberine found in different Berberis species have also been described [9].

*Berberis baluchistanica* Ahrendt is wild medicinal plant locally known as Zralag in Pashto, Archin in Brahvi, and Korae in Balochi languages. It is endemic to Balochistan and belongs to family *Berberidaceae*. It is an evergreen shrub three meter tall with red brown to red stem and thick rigid leaves, harboring yellow color flowers between the months of March to May. The plant is distributed in Harboi, Kalat, and Zarghun area of Quetta and Ziarat [10]. This medicinal plant is considered as nontoxic and used as decoction or powder form. Due to the presence of berberine, the plant is utilized locally to cure different diseases like cold, cough, fever, internal injury, diseases of eyes, kidney stones removal, and wound [10, 11]. Berberisinol, oleanolic acid, berberine, gallic acid, 8-oxoberberine, palmatine, polyphenols, and vitamins were obtained with its notable antioxidant and antimicrobial [12]. Previously, [13] analyzed that the extract of root has strong antibacterial effects against a variety of pathogenic bacteria. The presence of these valuable components makes this plant medicinally important. Though the plant is generally used in local medicines, limited work has been reported on its phytochemicals and pharmacological activities. In recent years, much consideration has been paid to evaluate the bioactive components of medicinal plants, their chemical nature, antioxidant, and antimicrobial potentials. Similar studies are needed to investigate the curative potential of *Berberis baluchistanica* an indigenous plant for its actual health application and potential assessments. Hence, the current study was aimed at analyzing the bioactive components, total phenolics and flavonoids contents, antioxidant potential, and antimicrobial power of crude ethanolic extracts of root of *Berberis baluchistanica* Ahrendt. Furthermore, the biologically active compounds of the root extract were also analyzed by GC-MS for bioactive chemical profiling.

The article "High Throughput Screening for Bioactive Components of Berberis baluchistanica Ahrendt Root and Their Functional Potential Assessment" was published in 2022. Journal: Biomed Res Int.

## 2. Materials and Methods

### 2.1. Collection of Plant Samples

The plant was collected from district Ziarat Balochistan, identified by taxonomists Dr. Shazia Saeed Assistant Professor Botany and banked in the Herbarium, Department of Botany University of Balochistan Quetta, Pakistan.

### 2.2. Sample Preparation

The root was separated from the plant, washed off to make it dust and contaminations free, and was dried at room temperature for 3-4 weeks consecutively in controlled environment. Electrical grinder was used to crushed the root into powdered and stored in desiccators at room temperature for further analysis [14].

### 2.3. Extraction of Compounds

One liter ethanol was used for the maceration extraction of root fine powder (100 g) keeping 1 : 10 ratio following [14]. Light exposures were avoided during the maceration process by doing the experiments in dark room. The mixture was shaken with specific frequency for better extraction of compounds. Whatman filter No. 1 filter paper was used to filter the ethanolic mixture. The mixture was dried in rotary evaporator (LEV400T-L), and the thick extracts was used for biological and functional activities determination.

### 2.4. Bioactive Component Analysis

The ethanolic extract of root was analyzed for the identification and occurrence of alkaloids, tannins, glycosides, anthraquinones, saponins, flavonoids, coumarin, quinones, steroids, terpenoids, and phlobatannins through phytochemical analysis following the standard methods [14, 15].

### 2.5. Total Phenolic Content

For total phenolic contents of root extract, the Folin Ciocalteu reagent method described by [16] was followed with slight modification. A stock solution (1 mg/mL) of dried crude plant extract was diluted with deionized water to make 1, 0.5, 0.25, 0.125, and 0.0625 mg/mL. For extract, 0.5 mL was mixed with freshly prepared (2 mL) Folin Ciocalteu reagent and mixed properly followed by 5 min incubation at room temperature and further neutralized with 2 mL 10% Na_2_CO_3_ and mixed followed by 30 min incubation. The absorbance was calculated at 750 nm using T60 UV-visible spectrophotometer (PG, UK). Ethanol (95%) was used as blank. For the quantification of the extract, a calibrations curve was made from diverse dilutions of gallic acid. The findings were articulated as milligram of gallic acid equivalents (GAE)/g of sample dried weight.

The article "High Throughput Screening for Bioactive Components of Berberis baluchistanica Ahrendt Root and Their Functional Potential Assessment" was published in 2022. Journal: Biomed Res Int.

### 2.6. Total Flavonoid Contents

Aluminum chloride colorimetric method as explained by [17] was used for the total flavonoids content determination. Simply 0.5 mL (1 mg/mL) of the extract was mixed up with 95% ethanol and 0.5 mL NaNO_2_ (5%) solution, 0.1 mL (10% *w*/*v*, 0.1 mL) of AlCl_3_.6H_2_O, (0.5 mL of 1 M) NaOH and 2 mL of de-ionized water was added and incubated for 40 min at 25°C. Absorbance at 415 nm was measured by using T60 UV-visible spectrophotometer (PG, UK) against blank. Quantifications were made on the basis of a standard curve from different concentrations of quercetin. Results were denoted as mg quercetin equivalents per gram of sample (mg QE/g sample). Each step was carried in triplicates.

### 2.7. Protein Determination by Lowry's Method

Lowry's method was used for protein contents analysis [18]. Simply 4 mL of reagent 1 [2%Na_2_CO_3_ (48 mL) in 0.1 N NaOH + 1%KNaC_4_H_4_O_6_.4H_2_O (1 mL) + 0.5%CuSO_4_.5H_2_O (1 mL)] was added to 0.5 mL of each extract followed by 15 min incubation. After that, 0.5 mL of freshly prepared reagent 2 (2 mL Folin Ciocalteu reagent, 4 mL water with 1 : 2 ratio) was mixed rapidly and incubated for 30 min in dark. Standard reagent Bovine Serum Albumin was used for standard curve preparing and deionized water as blank. Subsequently, the absorbance of the standard solutions and sample extract was calculated at 660 nm. The quantification was completed in triplicate, and the amount of protein was mentioned as mg BSAE/g of sample [19].

### 2.8. DuBois Carbohydrate Assay

Carbohydrates were estimated by phenol sulphuric reagent method. Phenol 80% (0.05 mL) was added to extract (1 mL), and then, concentrated H_2_SO_4_ (5 mL) was added and kept for 10 min. The mixture was put in a water bath at 25° to 30° C for 10 to 20 minutes, and change in color was observed. The absorbance of the characteristic yellow orange color was measured at 510 nm. Deionized water was used as blank, and glucose was used as a standard. The results were mentioned as mg GE/g [19].

The article "High Throughput Screening for Bioactive Components of Berberis baluchistanica Ahrendt Root and Their Functional Potential Assessment" was published in 2022. Journal: Biomed Res Int.

### 2.9. Quantitative Assay for DPPH Free Radical Scavenging Activity

The hydrogen donating capability of root extract was carried out in the presence of DPPH stable radical. Different concentrations (1-0.0625 mg/mL) of root extract were made from stock solution, and 0.1 mM DPPH solution (0.5 mL) (for making DPPH 0.1 mM, add 0.0039432 g of DPPH in absolute ethanol 100 mL) was mixed up with 50 *μ*L of the extract. The reaction mixture was shaken and incubated at room temperature for reaction at dark place for 30 min using ascorbic acid as standard. Decolorization of DPPH was observed by measuring the decrease in absorbance at 517 nm. The ethanol, ascorbic acid, and DPPH solution without plant extract were used as a blank, standard, and control correspondingly [14, 17].

The following equation was used for % inhibition calculation:

(1) $$\begin{array}{c} \%\text{ inhibition of DPPH}=\frac{\left(\text{AC}-\text{AS}\right)}{\text{AC}}\times 100. \end{array}$$

Here, AC is absorbance of control (DPPH), and AS is extract absorbance.

The IC_50_ values describe the concentration of sample extract used for scavenging 50% of the DPPH free radicals by characterizing the antioxidant ability of the extracts. The relationship curve was made by plotting the scavenging activities against different concentrations of extract and expressed in mg/mL.

### 2.10. Ferric Reducing Antioxidant Power (FRAP) Assay

For the FRAP assay, the procedure from [20] was followed with little modifications. Stock solution comprised of acetate buffer (300 mM) with pH 3.6, TPTZ (10 mM) solution, prepared in HCL (40 mM), and ferric chloride hexahydrate (20 mM) solution. The solution was made by mixing acetate buffer (25 mL), TPTZ solution (2.5 mL), and ferric chloride hexahydrate solution (2.5 mL) with 10 : 1 : 1 (*v*/*v*), respectively. Briefly, 0.5 mL of the extract (1 mg/mL) was taken in test tubes and 2 mL of FRAP solution and 1 mL distilled water was added. The extract was allowed to react with FRAP solution in the dark for 30 minutes. Absorbance of the colored product was checked at 593 nm. Distilled water was taken as blank, and FeSO_4_ was taken as standard. The analysis was carried out in triplicates for the extract, and % reduction was determined by the following equation:

(2) $$\begin{array}{c} \text{FRAP }\%\text{ Reduction}=\frac{\left(\text{AC}-\text{AS}\right)}{\text{AC}}\times 100, \end{array}$$

where AC is the absorbance of control, and AS is the absorbance of the extract.

### 2.11. Antibacterial Activity

The antibacterial potential of *Berberis baluchistanica* root extract was evaluated by using agar well diffusion method. Fresh sterile Mueller Hinton agar was inoculated with the target bacterial strains *Klebsiella pneumoniae*, *Pseudomonas aeruginosa*, *Staphylococcus aureus*, *Escherichia coli*, and *Salmonella typhi*. Wells were made through 6 mm sterilized cork borers in the plates and extracts dissolved in dimethyl sulfoxide (100 *μ*L) were added into the agar wells. Dimethyl sulfoxide and doxycycline (DO 30 *μ*g) were used as negative and positive controls. The results were observed after 16-24 h of incubation at 37°C, diameter of the inhibition zones was measured in millimeter (mm) [21].

The article "High Throughput Screening for Bioactive Components of Berberis baluchistanica Ahrendt Root and Their Functional Potential Assessment" was published in 2022. Journal: Biomed Res Int.

### 2.12. Gas Chromatography-Mass Spectrometry Analysis

The GC-MS study was executed using a (Shimadzu GC-MS QP2020) gas chromatograph mass spectrometer supplied with an HP-INNOWAX capillary column (30 m length × 0.25 mm id 0.25 mm film thickness) (PaloAlto, CA, USA). The mass spectrum was obtained by electron ionization at 70 eV with a mass scan mode range of 35-500 amu (atomic mass units). The carrier gas helium was used at a flow rate of 1 mL/min, about 2 *μ*L volume of the sample was injected, and the injection temperature was 255°C with a split ratio 1 : 10. The oven temperature for the GC was initially organized at 50°C for 5 min then increased at the rate of 250°C at 5°C/min and finally to 300°C at 5°C/min for 10 min. The start temperature was 50°C and increased at the rate of 8°C/min to 250°C followed by 5°C/min till 300°C. The identification and composition of the targeted compounds were validated by comparing their mass spectral record with those of NIST 14 and 14 s (National Institute of Standards and Technology) Libraries. Mass spectrum was used to identify the name, molecular formula, molecular weight, and structure of the components.

### 2.13. Statistical Analysis

The measured data in each experiment comprised of 3 replications and the results were expressed as the average ± standard deviations (SD). The magnitude of the means, standard curve, and standard deviations were calculated by using MS Excel 2010 Software.

## 3. Results

### 3.1. Phytochemical Analysis

The phytochemical evaluation in root of *Berberis baluchistanica* indicated the presence of alkaloids, cardiac glycoside, anthraquinones, saponins, tannins, flavonoids, coumarin, steroids, and terpenoids. However, quinones and phlobatannins were not present in root (Table 1).

### 3.2. Phenolic Contents

Total phenolic contents of *Berberis baluchistanica* root extract were evaluated by Folin Ciocalteu method by using gallic acid as standard. Total phenolic content of the extract was determined from the regression equation and expressed as milligram gallic acid equivalents (GAE) per gram in dry weight of sample. TPC value was 19.897 ± 4.8141 mg GAE/g for root extract (Table 2).

The article "High Throughput Screening for Bioactive Components of Berberis baluchistanica Ahrendt Root and Their Functional Potential Assessment" was published in 2022. Journal: Biomed Res Int.

### 3.3. Flavonoid Contents

Total flavonoid content was determined, and results were calculated from the calibration curve and expressed as mg quercetin equivalents (QE) per gram of sample in dry weight. The total flavonoids in root extract were 12.9876 ± 0.8388 mg QE/g as presented in (Table 2).

### 3.4. Total Protein and Carbohydrates

Total protein contents in root of *Berberis baluchistanica* were calculated by Lowry's method ,and the absorbance values were obtained at various concentrations of BSA for the construction of calibration curve. Total proteins of the extract were 4.675 ± 0.1696 (mg BSAE/g) for root extract (Table 2).

Carbohydrate estimation was carried out by phenol sulphuric reagent method using glucose as standard. A linear trend was observed between the glucose standards concentration and the absorbance at 510 nm. The carbohydrate contents in root extract were 3.696 ± 0.2958 (mg GE/g) as presented in (Table 2).

### 3.5. Quantitative Assay for DPPH Free Radical Scavenging Activity

The hydrogen donating capability of the root extract of *Berberis baluchistanica* was determined in the presence of DPPH stable radical, and their reducing potential was calculated on the basis of their concentration showing 50% inhibition that is the concentration of extract needed to scavenge 50% DPPH free radicals. The results were obtained by the linear regression equation formed by the concentration of extract against their % scavenging ability. In present study, the DPPH radical scavenging activity was recorded with IC_50_ = 1.125 mg/mL in comparison with the standard ascorbic acid having IC_50_ = 0.325 mg/mL as shown in (Table 3). The radical scavenging activity increased with increased in concentration is shown in (Table 4 and Figure 1(a)).

### 3.6. Ferric Reducing Antioxidant Power Assay

The antioxidant capacity of *Berberis baluchistanica* root extract was determined by ferric reducing antioxidant power (FRAP) assay. Results were expressed on the basis of their concentration providing 50% inhibition (IC_50_) that is the concentration of extract required to reduce Fe3+ into Fe2+. The results were obtained by the linear regression equation formed by the concentrations of extracts against their percent of reducing ability. Obtained results showed that the extract has FRAP % reduction activity with IC_50_ = 0.912 mg/mL as presented in Table 3. The higher IC_50_ value indicates lower antioxidant potential and same for ferric reducing activity. In comparison with the standard having IC_50_ value 0.472 mg/mL, the root extract showed lowest antioxidant potential with higher IC_50_ value 0.912 mg/mL. The current findings revealed that the radical scavenging activity of the extract increased with increase in concentration as shown in Table 4 and Figure 1(b).

The article "High Throughput Screening for Bioactive Components of Berberis baluchistanica Ahrendt Root and Their Functional Potential Assessment" was published in 2022. Journal: Biomed Res Int.

### 3.7. Antibacterial Activity

The root extract of the *Berberis baluchistanica* plant was evaluated for its antibacterial properties against different bacteria. The diameter of the inhibition zones against *Escherichia coli*, *Pseudomonas aeruginosa*, *Staphylococcus aureus*, *Klebsiella pneumoniae*, and *Salmonella typhi* were 23.14 ± 1.16, 13.38 ± 0.41, 20.21 ± 0.06, 7 ± 0.01, and 14.84 ± 1.06. The extract was found to be active against selected bacteria except *Klebsiella pneumoniae* that showed minimum inhibition, and the activity has been shown in (Figure 2) comparing to the positive control applied in the study. The negative control DMSO was found inactive against all the targeted bacteria.

### 3.8. GC-MS Analysis

The GC-MS analysis of root extract is given in (Table 5), and the characteristic chromatogram is shown in (Figure 3). The extract is found to contain more than 70 different compounds belonging to different chemical classes with high therapeutic potential. The major compounds included 4-hydroxy-3-(4-hydroxy-3-nitrocinnamoyl)-, 1,3-dioxane-5,5-dimethanol, 2-methyl-, 4-[5-(4-fluoro-phenyl)-tetrazol-2-yl]-butyramide, bicyclo -3-en-2-one, 3,8-dihydroxy-1-methoxy-7-, allyloxydi(tert-butyl)silane, imidazo[1,2-a]pyridin-2(3H)-one, 8-(dimethylamino)-1-hydroxynaphthalene-2-carbonitrile, bicyclo[2.2.1]hept-5-ene-2-carboxylic acid, 7,7-dimethoxy-, 4-allyl-3-(dimethylhydrazono)-2-methylhexane-2, 5-diol, carbonic acid, 2-chloroethyl 2-pentyl ester, carbonic acidbut-3-yn-1-yl octyl ester, acetonitrile, 2,2′-iminobis-, acetic acid, cyano-, 2-hexynoic acid, pyrimidin-4(3H)-one, 2-amino-6-hydroxy-5-nitro-, 3-chlorophenyl pent-4-en-2-yl ester, isoquinoline, decahydro-, 1-nitrobiuret, 6-chloromethyl-N,N-dimethyl-[1,3,5]triazine-2,4-diamine, methyl 3-hydroxyoctadecanoate, TMS derivative, cephaloridine, 3,6,9,12-tetraazatetradecane-1,14-diamine, N(2),N(6)-bis(dimethylaminomethylene)lysine, cholestan-3-ol, TMS derivative, 3-methyl-4-nitro-5-(1-pyrazolyl)pyrazole, 2-naphthalenecarboxylic acid, 4,4′-methylenebis[3-methoxy-, p-undecyloxybenzoic acid methyl ester, 4-penten-2-ynylamine, N,N,4-trimethyl-, acetamide, N-(aminocarbonyl)-2-chloro-, piperazine, 2-methyl-, cyclopentane, 1-methyl-3-(2-methyl-2-propenyl)-, ethanone, 1-(4-pyridinyl)-, oxime, thiourea, dimethylaminomethyl, histamine-2-carboxylic acid, 9,12-octadecadienoic acid (Z,Z)-, pentanedioic acid, 2,4-dimethyl-, dimethyl ester, bis(sec-butoxo)(methyl)oxovanadium, methyl 4-(2,4-dinitrophenylhydrazono) valerate, dihydroartemisinin, 6-deshydro-5-deshydroxy-3-deoxy, lavandulyl butyrate, butanoic acid, 2,3-dichloro-, silane, (dotriacontyloxy)trimethyl-, 6-methyl-1-(2-thenylidene)furo[3,4c]pyridine, N-heptyl-2-(2-hydroxyethoxy)-N methylpropionamide, urea, N,N′-diethyl-, erythritol, acetamide, 2-chloro-N-1H-purin-6-yl-benzamide, 4-methoxy-N-[4-(1-methylcyclopropyl)phenyl]-,glycylglycine ethyl ester, 4-methyl-2,4-bis(p-hydroxyphenyl)pentene, (3-methylthiopropylideneamino)acetonitrile, androst-5-en-17-one, 16-(1,1-dimethylethyl)-3-hydroxy-, aminohippuric acid, 3TMS derivative, 7-methyl-6,8 bis(methylthio) pyrrolo [1, 2] pyrazine, cyclotetrasiloxane, octamethyl-,pentanedioic acid, 3,3-dimethyl-, dimethyl ester, N,N-dimethylsuccinamic acid, silicic acid, diethyl bis(trimethylsilyl)ester, p-phenylenediamine, N,N-dimethyl-N′-,benzestrol, 2TMS derivative, 6-chlorohexanoic acid, 4-cyanophenyl ester, pentasiloxane, dodecamethyl-,cyclotrisiloxane, hexamethyl-, 4-methyl-2,4-bis(p-hydroxyphenyl)pent-1-ene, trisiloxane, 1,1,3,3,5,5-hexamethyl-, cyclooctyl N,N-di isopropyl phosphoramidocyanidate, N-trifluoroacetyl-3-methoxytyramine, cyclotrisiloxane, hexamethyl-, 4-methyl-2,4-bis (p-hydroxyphenyl) pentene, 6-methoxypurine, and TBDMS derivative. These identified compounds are known to have several pharmacological potentials.

The article "High Throughput Screening for Bioactive Components of Berberis baluchistanica Ahrendt Root and Their Functional Potential Assessment" was published in 2022. Journal: Biomed Res Int.

## 4. Discussion

The current study was conducted to analyze the bioactive components and antimicrobial activity of root extract of the *Berberis baluchistanica* plant. Different bioactive compounds such as alkaloids, tannins, cardiac glycosides, anthraquinones, saponins, flavonoids, phenolics, coumarin, steroids, and terpenoids were detected. Many compounds such as phenolics, berberine, alkaloids, pakistanamine, gallic acid, and flavanols have already been reported [11, 13]. All the identified compounds are known to be biologically active possessing antibacterial, antifungal, antiviral, antiparasitic, and antioxidant potentials [10, 22].

The presence of these phytochemicals provides credibility to its use by the local community, and the discovery of new drugs will lead to understand the therapeutic effects of valuable compounds in medicinal plants [23].

Medicinal plants possess phenolic and flavonoid contents that are known to have antimicrobial, antispasmodic, antitumor, antioxidant, anti-inflammatory, and antidepressant activities [23]. Phenolic compounds are good reducing agents and are capable for scavenging of free radicals [24] and also regulate cell division, growth, and metabolic pathways in plants [22]. Flavonoid also reduces a wide range of enzymes like alkaline phosphatase, hyaluronidases, hydrolases, arylsulphatase, cAMP phosphodiesterase, lipase, *α*-glucosidase, and kinases [25]. The higher phenolic content supports the antioxidant property of plants. Therefore, the occurrence of total phenolics and flavonoid contents was investigated (Table 4).

The article "High Throughput Screening for Bioactive Components of Berberis baluchistanica Ahrendt Root and Their Functional Potential Assessment" was published in 2022. Journal: Biomed Res Int.

Previously, the total phenolic contents of *Berberis baluchistanica* whole plant were determined by using different fractions [26]. The obtained values of TPC and TFC in current study were propositionally lower than previously reported [26]. Recently, phenolic and flavonoids contents in bark extract were reported as 48.2 mg GAE/g and 141.3 mg QE/g [10]. These variations could arise from variations in plant species, genetic backgrounds, growing conditions, environmental factors, and agronomic practices polarity of the solvents [27].

The phenolic and flavonoid contents are responsible for the biological effects of the crude extract. Flavonoids are highly efficient in scavenging of oxidizing molecule, including different free radicals involved in various diseases [28]. Phenolic contents contribute the stress tolerance in plants. Extracts of herbs, vegetables, fruits, and grains being rich in phenolics are increasingly used in the food industries for their antioxidative potentials and medical advantages. Similarly, flavonoid suppresses the formation of reactive oxygen involved in production of free radicals and scavenging of reactive species for antioxidant defense.

The DPPH assay is considered as one of the most valid used tools to identify the scavenging potential of free radical by plant extracts. The IC_50_ value is basically concentration of substrate which inhibits 50% of DPPH radicals. In the current study, the obtained results of DPPH radical scavenging activity were higher than the ethyl acetate soluble fraction IC_50_ value (15.96 ± 1.5 *μ*g/mL) of the whole plant of *Berberis baluchistanica* reported by [26]. Current findings were higher than the recently reported antioxidant activity IC_50_ (52.86 *μ*g/mL) of CME of *Berberis baluchistanica* [12]. The lower IC_50_ value indicates higher antioxidant potential and same for radicals scavenging activity. The antioxidant power of plants extracts is generally associated with the concentration of phenolic and flavonoid compounds present in the sample. Higher quantity of polyphenols and flavonoids describes the higher antioxidant activity [14]. Literature reveals that berberine an alkaloid and berberisinol flavones obtained from Berberis species exhibit antioxidant potential. Berberine and berberisinol also present in *Berberis baluchistanica* [29] might be a causative factor for hydrogen donor capacity of *Berberis baluchistanica* ethanolic root extract.

The article "High Throughput Screening for Bioactive Components of Berberis baluchistanica Ahrendt Root and Their Functional Potential Assessment" was published in 2022. Journal: Biomed Res Int.

FRAP % reduction activity was done to measure the antioxidant capacity of *Berberis baluchistanica* root extract against reactive oxygen species. Antioxidants have capability to give electrons and reduce Fe3+ into Fe2+. The complexes of Fe2+ and tripyridyltriazine give an intense blue color with high absorbance at wavelength of 593 nm. The antioxidant capacity of the extracts was related to the IC_50_ values. The higher IC_50_ values indicate lower reducing activity or lower antioxidant potential. The present study revealed that the ethanolic root extract exhibited lower FRAP % reduction with IC_50_ (0.912 mg/mL). Obtained results were in conformity with previous data [26]. Phenolic and flavonoids have made significant antioxidant power as they act as suitable scavenging agents. According to [6], the total antioxidant activity was directly related to phenolic compounds. Moreover, comparing our results of antioxidant activity showed strong correlation between DPPH and ferric reducing antioxidant power assay. Results revealed that total antioxidant activity of root extract is due to its higher association with antioxidant compounds such as phenols. Current findings were in agreement with previous reported literature [30].

The antibacterial potential of *Berberis baluchistanica* root extract was assessed by using agar well diffusion method. The extract showed effective antibacterial potential against bacterial strains of *Escherichia coli*, *Staphylococcus aureus*, *Pseudomonas aeruginosa*, *Klebsiella pneumoniae*, and *Salmonella typhi*. Gram negative bacteria, *Escherichia coli* proved to be the most sensitive with maximum zone of inhibition (23.14 ± 1.16) followed by *Staphylococcus aureus* (20.21 ± 0.06). Results revealed that all selected pathogens were susceptible to the extract except *Klebsiella pneumoniae* that turned out to be the most resistant strain and showed minimum inhibition. The results of current study were linked with the previously reported [10] and relatively higher than those found in literature [13]. However, [11] documented higher results. Recently, [12] reported the crude methanolic extract of *Berberis baluchistanica* against *Pseudomonas aeruginosa* (Gram negative bacterium) and *Micrococcus luteus* and *Bacillus subtilis* (gram positive strains) at three different concentrations. All concentrations were found with better inhibitory profile *Micrococcus luteus* 16.81, 17.93, and 20.22 mm and *Bacillus subtilis* and 12.18, 16.72, and 18.37 mm, respectively. Similar trends were observed with the previously documented results of other species of *Berberis* [23, 29, 31]. The results suggested that root extract is a powerful source of wide-ranging antimicrobial agent. The strong antibacterial effect of the obtained extract is probably due to the presence of secondary metabolites such as alkaloids, steroids, coumarin, saponins, and terpenoids and high contents of phenolics and flavonoids which seemed to be associated in nucleic acid biosynthesis inhibition and new metabolic practices [25].

The article "High Throughput Screening for Bioactive Components of Berberis baluchistanica Ahrendt Root and Their Functional Potential Assessment" was published in 2022. Journal: Biomed Res Int.

The total proteins and total carbohydrates contents were determined by Lowry's method and phenol sulphuric reagent method, respectively. Total proteins of the extract were 4.675 ± 0.1696 (mg BSAE/g) and carbohydrate contents in root extract were 3.696 ± 0.2958 (mg GE/g). Current results of protein and carbohydrates estimation of *Berberis baluchistanica* root extract showed that it contains a reasonable amount of proteins and carbohydrates, so root can be used as a natural source of low cost and easily available proteins and carbohydrates enriched food material for nutritional purposes. Current findings were in accordance with previous findings [32].

The results of the GC-MS analysis revealed that a total of 70 different known compounds belonged to different chemical classes were identified. The active principles of the identified compounds with their retention time, concentration (area %), molecular formula, and molecular weight are presented in Table 5. The representative chromatograms of the ethanolic root extract of *Berberis baluchistanica* are presented in Figure 3.

GC-MS study was executed to recognize the biologically active components present in root of *Berberis baluchistanica* due to the fact that the plant has many phytochemicals possessing several therapeutic activities. From the results, it was observed that 70 different compounds with the mass spectra have been identified. The results revealed that the detected compounds were as traces (below 0.5%). Among major compounds, 9,12-octadecadienoic acid (Z,Z)- is known to have anti-inflammatory, hypocholesterolemic, and antiarthritic property [19]. Recently, [33, 34] reported the strong antioxidant, anti-inflammatory, cytotoxicity, nematicidal, and antibacterial potential of hexadecanoic acid and pentanedioic acid methyl ester. Naphthalene is also reported to possess strong antioxidant, antifibrinolytic, and antimicrobial activity [19]. Strong antioxidant, anti-inflammatory, and cytotoxicity of acetamide were reported by [35]. Presence of silicic acid, diethyl bis(trimethylsilyl) ester in relatively higher quantity might be accountable for the biological strength of the extract against human pathogen [36]. Erythritol is a sweet antioxidant releases oxidative stress and has unique nutritional properties [37]. Some other significant medicinal compound p-andecyloxybenzoic acid methyl ester, benzamide, benzestrol, thiourea, and dimethylaminomethyl were also reported by the earlier workers [38–40]. The principle identified compounds in the sample are 4-hydroxy-3-(4-hydroxy-3-nitrocinnamoyl)-,1,3dioxane-5,5-dimethanol,2-methyl-bicyclooct-3-en-2-one,3,8-dihydroxy-1-methoxy-7-3,8-dihydroxy-1-methoxy-7, allyloxydi(tert-butyl)silane,7,7-dimethoxy-,5-diol, carbonic acid, 2-chloroethyl 2-pentyl ester, carbonic acid but-3-yn-1-yl octyl ester, acetonitrile, 2,2′-iminobis-, acetic acid, cyano-, 2-hexynoic acid, pyrimidin-4(3H)-one, 2-amino-6-hydroxy-5-nitro-, succinic acid, isoquinoline, decahydro-, 2-naphthalenecarboxylic acid, 4,4′-methylenebis[3-methoxy-, p-undecyloxybenzoic acid methyl ester, 4-penten-2-ynylamine, N,N,4-trimethyl-, acetamide, N-(aminocarbonyl)-2-chloro, piperazine,2-methyl-, cyclopentane, 1-methyl-3 (2-methyl-2-propenyl), cyclotrisiloxane, hexamethyl-, N-trifluoroacetyl-3-methoxytyramine, and methoxypurine derivative and were also present. GC-MS analysis of *Berberis baluchistanica* root extract showed a mixture of acetamides, glycosides, and methyl esters, and its derivatives that are known to have significant antioxidant, inflammatory, hypocholesterolemic and antiarthritic and cytotoxicity and antibacterial properties [41].

The article "High Throughput Screening for Bioactive Components of Berberis baluchistanica Ahrendt Root and Their Functional Potential Assessment" was published in 2022. Journal: Biomed Res Int.

## 5. Conclusion

The obtained results clearly showed that *Berberis baluchistanica* root extract is rich in bioactive compounds with strong antioxidant potential. The extract was found to have significant antimicrobial potential against different bacterial pathogens. The protein and carbohydrate estimation shows that it contains low cost and easily available proteins and carbohydrates enriched food material for nutritional purposes. GC-MS analysis established the existence of various bioactive compounds in root extract having the potential to act as antimicrobial, antioxidant, anti-inflammatory, cytotoxicity, and nematicidal substances. From this study, it can be concluded that the *Berberis baluchistanica* root may provide a potential source of medicines due to the presence of biologically active components with strong antioxidant and antibacterial activities.

## Figures and Tables

**Figure 1:** (a) Free radical scavenging activity (DPPH). (b) Ferrous reducing capacity (FRAP) of root ethanolic extract of *Berberis baluchistanica*, (■) represent standard, while (●) represent root sample. Ascorbic acid and ferrous sulfate (FeSO_4_) were used as a standard in DPPH and FRAP.

**Figure 2:** Antibacterial activity of *Berberis baluchistanica* root extract against various bacterial strains *E. coli* (*Escherichia coli*), *K. pneumoniae* (*Klebsiella pneumoniae*), *P. aeruginosa* (*Pseudomonas aeruginosa*), *S. aureus* (*Staphylococcus aureus*), and S. typhi (Salmonella typhi).

The article "High Throughput Screening for Bioactive Components of Berberis baluchistanica Ahrendt Root and Their Functional Potential Assessment" was published in 2022. Journal: Biomed Res Int.

**Figure 3:** GC-MS chromatograph of ethanolic root extract of *Berberis baluchistanica.*

**Table 1:** Phytochemical constituents of the *Berberis baluchistanica* root extracts.

S. no	Phytochemical test	Results
1.	Alkaloids	+ve
2.	Cardiac glycosides	+ve
3.	Tannins	+ve
4.	Steroids	+ve
5.	Terpenoids	+ve
6.	Flavonoids	+ve
7.	Saponins	+ve
8.	Coumarin	+ve
9.	Quinones	-ve
10.	Anthraquinones	+ve
11.	Phlobatannins	-ve

Note: +ve: present and –ve: absent.

**Table 2:** Total phenolic contents, total flavonoid contents, total protein, and carbohydrates.

Samples	Total phenolic (mg GAE/g) ± SD	Total flavonoid (mg QE/g) ± SD	Total proteins (mg BSAE/g) ± SD	Total carbohydrates (mg GE/g) ± SD
Root	19.897 ± 4.8141	12.9876 ± 0.8388	4.675 ± 0.1696	3.696 ± 0.2958

Results are expressed as Mean ± S.D for three readings.

**Table 3:** Estimated IC_50_ values of ethanolic root extract of *Berberis baluchistanica.*

Samples	DPPH assay (IC_50_ mg/mL)	FRAP assay (IC_50_ mg/mL)
Root	1.125	0.912
Ascorbic acid (standard)	0.325	**—**
FeSO_4_ (standard)	**—**	0.472

Ascorbic acid and FeSO_4_ = standard.

**Table 4:** DPPH percentage inhibitions and FRAP percent reduction of *Berberis baluchistanica* root extract at different concentration.

Concentrations in (mg/mL)	DPPH % inhibition	FRAP % reduction
1	44.91 ± 0.67	68.92 ± 0.81
0.5	36.43 ± 1.07	56.72 ± 0.24
0.25	17.86 ± 0.94	41.13 ± 1.01
0.125	12.47 ± 1.22	29.12 ± 0.56
0.0625	0.10 ± 0.073	12.01 ± 0.63

**Table 5:** The major bioactive compounds analyzed in the ethanolic root extract of *Berberis baluchistanica* by GCMS analysis.

S.#	Retention time (min)	Area (%)	Name of the compound	Mol. formula	Mol. Weight
1.	4.728	0.15	4-Hydroxy-3-(4-hydroxy-3-nitrocinnamoyl)-	C_15_H_11_NO_7_	317
2.	4.855	0.08	1,3-dioxane-5,5-dimethanol, 2-methyl-	C_7_H_14_O_4_	162
3.	5.559	0.47	4-[5-(4-Fluoro-phenyl)-tetrazol-2-yl]-butyramide	C_11_H_12_FN_5_O	249
4.	6.255	0.25	Bicyclo -3-en-2-one, 3,8-dihydroxy-1-methoxy-7-	C_21_H_24_O_7_	388
5.	6.523	0.17	Allyloxydi(tert-butyl)silane	C_11_H_23_OSi	199
6.	7.531	0.08	Imidazo[1,2-a]pyridin-2(3H)-one	C_7_H_6_N_2_O	134
7.	8.045	0.14	8-(Dimethylamino)-1-hydroxynaphthalene-2-carbonitrile	C_13_H_12_N_2_O	212
8.	9.737	0.25	Bicyclo[2.2.1]hept-5-ene-2-carboxylic acid, 7,7-dimethoxy-	C_10_H_14_O_4_	198
9.	10.834	0.09	4-Allyl-3-(dimethylhydrazono)-2-methylhexane-2, 5-diol	C_12_H_24_N_2_O_2_	228
10.	11.628	0.11	Carbonic acid, 2-chloroethyl 2-pentyl ester	C_8_H_15_ClO_3_	194
11.	12.961	0.02	Carbonic acidbut-3-yn-1-yl octyl ester	C_13_H_22_O_3_	226
12.	13.083	0.07	Acetonitrile, 2,2′-iminobis-	C_4_H_5_N_3_	95
13.	13.143	0.14	Acetic acid, cyano-	C_3_H_3_NO_2_	85
14.	14.409	0.1	2-Hexynoic acid	C_6_H_8_O_2_	112
15.	14.524	0.11	Pyrimidin-4(3H)-one, 2-amino-6-hydroxy-5-nitro-	C_4_H_4_N_4_O_4_	172
16.	16.05	0.1	3-chlorophenyl pent-4-en-2-yl ester	C_15_H_17_ClO_4_	296
17.	16.685	0.2	Isoquinoline, decahydro-	C_9_H_17_N	139
18.	17.821	0.2	1-Nitrobiuret	C_2_H_4_N_4_O_4_	148
19.	18.09	0.1	6-Chloromethyl-N,N-dimethyl-[1,3,5]triazine-2,4-diamine	C_6_H_10_ClN_5_	187
20	19.025	0.02	Methyl 3-hydroxyoctadecanoate, TMS derivative	C_22_H_46_O_3_Si	386
21.	20.409	0.1	Cephaloridine	C_19_H_17_N_3_O_4_S_2_	415
22.	20.554	0.1	3,6,9,12-Tetraazatetradecane-1,14-diamine	C_10_H_28_N_6_	232
23.	21.79	0.08	N(2),N(6)-Bis(dimethylaminomethylene)lysine	C_13_H_26_N_4_O_2_	270
24.	21.445	0.08	Cholestan-3-ol, TMS derivative	C_30_H_56_OSi	460
25.	22.688	0.15	3-Methyl-4-nitro-5-(1-pyrazolyl)pyrazole	C_7_H_7_N_5_O_2_	193
26.	22.963	0.06	2-Naphthalenecarboxylic acid, 4,4′-methylenebis[3-methoxy-	C_25_H_20_O_6_	416
27.	24.365	0.3	p-Undecyloxybenzoic acid methyl ester	C_19_H_30_O_3_	306
28.	25.712	0.17	4-Penten-2-ynylamine, N,N,4-trimethyl-	C_8_H_13_N	123
29.	26.77	0.12	Acetamide, N-(aminocarbonyl)-2-chloro-	C_3_H_5_ClN_2_O_2_	136
30.	27.49	0.1	Piperazine, 2-methyl-	C_5_H_12_N_2_	100
31.	28.31	0.16	Cyclopentane, 1-methyl-3-(2-methyl-2-propenyl)-	C_10_H_18_	138
32.	28.404	0.16	Ethanone, 1-(4-pyridinyl)-, oxime	C_7_H_8_N_2_O	136
33.	29.301	0.09	Thiourea, dimethylaminomethyl	C_4_H_11_N_3_S	133
34.	29.865	0.12	Histamine-2-carboxylic acid	C_6_H_9_N_3_O_2_	155
35.	30.364	0.03	9,12-Octadecadienoic acid (Z,Z)-	C_21_H_40_O_2_Si	352
36.	32.825	0.07	Pentanedioic acid, 2,4-dimethyl-, dimethyl ester	C_9_H_16_O_4_	188
37.	33.235	0.06	Bis(sec-butoxo)(methyl)oxovanadium	C_9_H_21_O_3_V	228
38.	34.605	0.19	Methyl 4-(2,4-dinitrophenylhydrazono) valerate	C_12_H_14_N_4_O_6_	310
39.	35.223	0.06	Dihydroartemisinin, 6-deshydro-5-deshydroxy-3-deoxy	C_15_H_22_O_3_	250
40.	35.725	0.07	Lavandulyl butyrate	C_14_H_24_O_2_	224
41.	36.241	0.12	Butanoic acid, 2,3-dichloro-	C_4_H_6_Cl_2_O_2_	156
42.	36.837	0.1	Silane, (dotriacontyloxy)trimethyl-	C_35_H_74_OSi	538
43.	36.935	0.11	6-Methyl-1-(2-thenylidene)furo[3,4c]pyridine	C_8_H_10_ClNO_2_	187
44.	37.53	0.2	N-Heptyl-2-(2-hydroxyethoxy)-N-methylpropionamide	C_13_H_27_NO_3_	245
45.	37.265	0.2	Urea, N,N′-diethyl-	C_5_H_12_N_2_O	116
46.	37.392	0.17	Erythritol	C_4_H_10_O_4_	122
47.	37.892	0.19	Acetamide, 2-chloro-N-1H-purin-6-yl-	C_7_H_6_ClN_5_O	211
48.	38.91	0.27	Benzamide, 4-methoxy-N-[4-(1-methylcyclopropyl)phenyl]-	C_18_H_19_NO_2_	281
49.	38.121	0.14	Glycylglycine ethyl ester	C_6_H_12_N_2_O_3_	160
50.	38.215	0.15	4-Methyl-2,4-bis(p-hydroxyphenyl)pentene	C_24_H_36_O_2_Si_2_	412
51.	38.395	0.13	(3-Methylthiopropylideneamino)acetonitrile	C_6_H_10_N_2_S	142
52.	39.985	0.2	Androst-5-en-17-one, 16-(1,1-dimethylethyl)-3-hydroxy-,	C_23_H_36_O_2_	344
53.	40.2	0.14	Aminohippuric acid,3TMS derivative	C_18_H_34_N_2_O_3_Si_3_	410
54.	40.58	0.24	7-Methyl-6,8 bis(methylthio) pyrrolo [1, 2] pyrazine	C_10_H_12_N_2_S_2_	224
55.	40.82	0.18	Cyclotetrasiloxane, octamethyl-	C_8_H_24_O_4_Si_4_	296
56.	40.151	0.23	Pentanedioic acid, 3,3-dimethyl-, dimethyl ester	C_9_H_16_O_4_	188
57.	41.006	0.34	N,N-Dimethylsuccinamic acid	C_6_H_11_NO_3_	145
58.	41.86	0.25	Silicic acid, diethyl bis(trimethylsilyl)ester	C_10_H_28_O_4_Si_3_	296
59.	41.106	0.18	p-Phenylenediamine, N,N-dimethyl-N′-	C_11_H_11_F_5_N_2_O	282
60.	41.148	0.27	Benzestrol, 2TMS derivative	C_26_H_42_O_2_Si_2_	442
61.	42.295	0.27	6-Chlorohexanoic acid, 4-cyanophenyl ester	C_13_H_14_ClNO_2_	251
62.	42.889	0.45	Pentasiloxane, dodecamethyl-	C_12_H_36_O_4_Si_5_	384
63.	43.25	0.24	Cyclotrisiloxane, hexamethyl-	C_6_H_18_O_3_Si_3_	222
64.	43.915	0.44	4-Methyl-2,4-bis(p-hydroxyphenyl)pent-1-ene	C_24_H_36_O_2_Si_2_	412
65.	44.194	0.33	Trisiloxane, 1,1,3,3,5,5-hexamethyl-	C_6_H_20_O_2_Si_3_	208
66.	44.423	0.27	Cyclooctyl N,N-di isopropyl phosphoramidocyanidate	C_15_H_29_N_2_O_2_P	300
67.	45.865	0.28	N-Trifluoroacetyl-3-methoxytyramine,	C_17_H_28_F_3_NO_3_Si_2_	407
68.	46.145	0.36	Cyclotrisiloxane, hexamethyl-	C_6_H_18_O_3_Si_3_	222
69.	46.456	0.48	4-Methyl-2,4-bis (p-hydroxyphenyl) pentene	C_24_H_36_O_2_Si_2_	412
70.	50.655	0.13	6-Methoxypurine, TBDMS derivative	C_12_H_20_N_4_OSi	264

The article "High Throughput Screening for Bioactive Components of Berberis baluchistanica Ahrendt Root and Their Functional Potential Assessment" was published in 2022. Journal: Biomed Res Int.

## Data Availability

Most of the data is part of the manuscript, and the remaining data will be made available on reasonable request.
